The article "Research on the Behavior Evolution of Interest Groups in Book Reverse Logistics" was published in 2022. Journal: Comput Intell Neurosci.

# Research on the Behavior Evolution of Interest Groups in Book Reverse Logistics

**DOI:** 10.1155/2022/3324312

**Published:** 2022-03-16

**Authors:** Shuihai Dou, Xianyang Su, Yanping Du, Yanming Tang, Lizhi Peng

**Affiliations:** ^1^Beijing Institute of Graphic Communication, Beijing, China; ^2^Zhenkunxing Industry Supermarket (Shanghai) Co., Ltd, Wuhan, China

## Abstract

With the gradual expansion of the book logistics market and the year-on-year increase in book publications, the incidence of book reverse logistics continues to increase, and the problem of book companies' inventory backlog has become increasingly prominent. To effectively alleviate the current backlog of book returns and exchanges, this paper constructs a two-party game model of “book publisher-book retailer,” analyzes the evolution process of book publishers and book retailers' participation strategies and the influence of parameter changes on stable strategies through theoretical analysis and numerical simulation, and draws the following conclusions. (1) Whether book publishers and book retailers choose to participate in the reverse logistics optimization of book returns and exchanges is closely related to their benefits and costs, and it also depends on whether the other party participates in the reverse logistics optimization of books. (2) When the cost of participating in book reverse logistics reaches a certain condition, the probability of both parties participating in the optimization is the greatest.

## 1. Introduction

With the rapid development of our country's society and economy, people's demand for spiritual culture is increasing day by day. The national inventory of books has increased substantially, reaching 6.64 billion books in 2014 [1]. At the same time, the incidence of reverse logistics in the book industry is the highest, generally around 30% [2]. In a certain period of time, the return rate of best-selling books will exceed 50% or even 60% [2]. Therefore, the problem of book backlog returns is no longer a disturbing factor affecting the economic development of the book industry but has become one of the leading factors that determine the economic development of the book industry. How to establish a good book reverse logistics between book publishers and book retailers to ensure the healthy and orderly development of the book logistics market is one of the key issues faced by managers and scholars in the industry.

To effectively alleviate the reverse logistics problem of book backlog inventory, Ma [3] established a book centralized inventory optimization model on the basis of analyzing the problems of book reverse logistics. Ning [4] built a collaboration mechanism with the focus on the green supply chain. Morgan [5] linked the sustainable supply chain management, resource input, and operational performance of reverse logistics and analyzed the sustainability of reverse logistics. Faustino et al. [6] introduced the concept of sustainability into reverse logistics and established an applicable reverse logistics process reference model. To accurately analyze the relationship of interest groups when book publishers and book retailers participate or not participate in the optimization of book reverse logistics, this paper consults relevant documents and sorts them out. Yi [7] and Xia [8] established a Stackelberg game model to analyze the group interest behavior of manufacturers and recyclers in reverse logistics. Ye [9] used evolutionary game theory to analyze the relationship between residents, government, and residents in the reverse logistics of waste sorting and recycling. Chen [10] established a game model to analyze the impact of recyclers on the supply chain under different parameter settings of the recycling mode. Wang [11] used game theory to establish a recycling decision model and analyzed product recycling strategies between manufacturers and retailers. Chen et al. [12], Shi et al. [13], and Ding et al. [14] used game theory to analyze the reverse logistics pricing of goods between manufacturers and recyclers.

The article "Research on the Behavior Evolution of Interest Groups in Book Reverse Logistics" was published in 2022. Journal: Comput Intell Neurosci.

Throughout the existing results, scholars at home and abroad have conducted little research on the evolution process and evolution law of the behavior of book reverse logistics interest groups, and they have rarely studied from the perspective of adaptation and evolution in reverse logistics scenarios to study the gradual change and evolution process of the book interest groups' participation strategies and behaviors by factors such as costs and benefits of reverse logistics. This paper takes book publishers and book retailers as research objects, explores the synergy between the two in the book reverse logistics optimization (hereinafter referred to as optimization), analyzes the behavioral evolutionary game of book publishers and book retailers participating in optimization decision making, and conducts numerical simulations to explore ways to effectively improve the active participation of both companies in book reverse logistics optimization, thereby reducing the inventory space occupied by the accumulation of books, reducing the resource waste of books, and making up for part of the vacancy in the study of the behavior evolution of the book reverse logistics interest groups.

## 2. Group Behavior Evolution Model of Book Publishers and Book Retailers

### 2.1. Scene Reappearance and Model Assumptions

In the book reverse logistics, because book publishers and book retailers consider complex and diverse factors when deciding whether to participate in the optimization of book reverse logistics, this paper makes the following assumptions without changing the nature of the problem:

1. Participants in the game: book publishers and book retailers are bounded rational subjects, and they will continue to learn and imitate the strategy choices of other individuals and improve their own revenue decisions, so strategies with higher returns will replace strategies with lower returns [15].
2. The strategic behavior of the game subject: both book publishers and book retailers can choose a positive strategy or negative strategy. The book publishers' strategy collection is (participation, non-participation), and the book retailers' strategy collection is (participation, non-participation).
3. The proportion of behavior strategy: assuming that in the initial stage of the evolutionary game, the proportion of book publishers participating in the optimization is *X*, then the proportion of not participating in the optimization is 1 − *X*, 0 ≤ *X* ≤ 1; the proportion of book retailers participating in the optimization is *Y*; then, the proportion of not participating in the optimization is 1 − *Y*, 0 ≤ *Y* ≤ 1.
4. Assume that the cost of book publishers choosing to participate in book reverse logistics optimization is greater than the cost of not participating in book reverse logistics optimization, that is, *C*_1_ > *S*_1_.
5. Assume that the cost of book retailers choosing to participate in book reverse logistics optimization is greater than the cost of not participating in book reverse logistics optimization, that is, *C*_2_ > *F*_2_.

The article "Research on the Behavior Evolution of Interest Groups in Book Reverse Logistics" was published in 2022. Journal: Comput Intell Neurosci.

Based on the above assumptions, this paper constructs a mixed strategy payment matrix between book publishers and book retailers, as shown in Table 1.

The parameters and explanations involved in the hybrid strategy payout matrix are as follows.

1. *α*_1_ and *α*_2_, respectively, represent the production and sales risk ratio of book publishers and book retailers. Production and sales risk refers to all the costs that book publishers and book retailers need to bear due to risks in the process of book reverse logistics, and *α*_1_ + *α*_2_ = 1.
2. *N* is all loss costs incurred in the process of book reverse logistics, including invisible losses such as negative impacts on the enterprise. Visible loss costs such as the backlog of unsalable books and excess shipping costs caused by reverse logistics and so on.
3. *C*_1_ and *C*_2_, respectively, represent the cost of book publishers and book retailers choosing to participate in book reverse logistics optimization, including the cost of purchasing new equipment and new technology, and so on.
4. *S*_1_ and *F*_2_, respectively, represent the cost of book publishers and book retailers choosing not to participate in book reverse logistics optimization, including the loading, unloading, handling, sorting, and other costs incurred in the process of book recycling.
5. *B*_1_ and *L*_2_, respectively, represent the revenue of book publishers and book retailers choosing to participate in book reverse logistics optimization.
6. *D*_1_ and *D*_2_, respectively, represent the revenue of book publishers and book retailers choosing not to participate in book reverse logistics optimization.

The article "Research on the Behavior Evolution of Interest Groups in Book Reverse Logistics" was published in 2022. Journal: Comput Intell Neurosci.

### 2.2. Establishment of Replication Dynamic Equation

According to the assumptions and the game payment matrix, this paper can get the expected returns *E*_*A*1_ and *E*_*A*2_ of book publishers choosing to participate in the strategy, non-participation strategy, and the average expected return ${\overset{-}{E}}_{A}$ of book publishers.

(1) $$\begin{array}{c} E_{A1}=Y\left(B_{1}-C_{1}-\alpha_{1}N\right)+\left(1-Y\right)\left(D_{1}-C_{1}-N\right)\\ =Y\left(B_{1}-D_{1}+N-\alpha_{1}N\right)+D_{1}-C_{1}-N,\\ E_{A2}=Y\left(D_{1}-S_{1}-N\right)+\left(1-Y\right)\left(D_{1}-S_{1}-N\right)=D_{1}-S_{1}-N,\\ {\bar{E}}_{A}=XE_{A1}+\left(1-X\right)E_{A2}. \end{array}$$

Then, we can get its dynamic replication equation *F*(*X*).

(2) $$\begin{array}{c} F\left(X\right)=\frac{\text{d}X}{\text{d}t}\\ =X\left(E_{A1}-{\bar{E}}_{A}\right)\\ =X\left(1-X\right)\left(E_{A1}-E_{A2}\right)\\ =X\left(1-X\right)\left[Y\left(B_{1}-D_{1}+N-\alpha_{1}N\right)+S_{1}-C_{1}\right]. \end{array}$$

In the same way, this paper can get the expected returns *E*_*B*1_ and *E*_*B*1_ of bookretailers choosing to participate in the strategy, non-participation strategy. The average expected return ${\bar{E}}_{B}$ of bookretailers, and the replication dynamic equation*F*(*Y*).

(3) $$\begin{array}{c} E_{B1}=X\left(L_{2}-C_{2}-\alpha_{2}N\right)+\left(1-X\right)\left(D_{2}-C_{2}\right)\\ =X\left(L_{2}-D_{2}-\alpha_{2}N\right)+D_{2}-C_{2},\\ E_{B2}=X\left(D_{2}-F_{2}\right)+\left(1-X\right)\left(D_{2}-F_{2}\right)\\ =D_{2}-F_{2},\\ {\bar{E}}_{B}=YE_{B1}+\left(1-Y\right)E_{B2},\\ F\left(Y\right)=\frac{\text{d}Y}{\text{d}t}\\ =Y\left(E_{B1}-{\bar{E}}_{B}\right)\\ =Y\left(1-Y\right)\left(E_{B1}-E_{B2}\right),\\ =Y\left(1-Y\right)\left[X\left(L_{2}-D_{2}-\alpha_{2}N\right)+F_{2}-C_{2}\right]. \end{array}$$

Thus, the replication dynamic equation, Jacobian matrix *J*, and the corresponding determinants and traces of the game system are obtained. For the sake of discussion below, let *β*_1_=*B*_1_ − *D*_1_+*N* − *α*_1_*N*+*S*_1_ − *C*_1_ and *β*_2_=*L*_2_ − *D*_2_ − *α*_2_*N*+*F*_2_ − *C*_2_.

(4) $$\begin{array}{c} \left\{\begin{array}{c} F\left(Y\right)=\frac{\text{d}Y}{\text{d}t}=Y\left(1-Y\right)\left[X\left(L_{2}-D_{2}-\alpha_{2}N\right)+F_{2}-C_{2}\right], \end{array}\right. \end{array}$$

(5) $$\begin{array}{c} J=\left[\begin{array}{cc} \frac{\partial F\left(X\right)}{\partial Y}\\ \frac{\partial F\left(Y\right)}{\partial X} & \frac{\partial F\left(Y\right)}{\partial Y} \end{array}\right] \end{array}$$

(6) $$\begin{array}{c} \det\left(J\right)=\left|\begin{array}{cc} \frac{\partial F\left(x\right)}{\partial y}\\ \frac{\partial F\left(y\right)}{\partial x} & \frac{\partial F\left(y\right)}{\partial y} \end{array}\right|=\frac{\partial F\left(x\right)}{\partial x}\cdot \frac{\partial F\left(y\right)}{\partial y}-\frac{\partial F\left(y\right)}{\partial x}\cdot \frac{\partial F\left(x\right)}{\partial y},\\ =\left(1-2X\right)\left[Y\left(B_{1}-D_{1}+N-\alpha_{1}N\right)+S_{1}-C_{1}\right]\cdot \left(1-2Y\right)\left[X\left(L_{2}-D_{2}-\alpha_{2}N\right)+F_{2}-C_{2}\right]\\ -Y\left(1-Y\right)\left(L_{2}-D_{2}-\alpha_{2}N\right)\cdot X\left(1-X\right)\left(B_{1}-D_{1}+N-\alpha_{1}N\right), \end{array}$$

(7) $$\begin{array}{c} \text{Tr}\left(J\right)=\frac{\partial F\left(x\right)}{\partial x}+\frac{\partial F\left(y\right)}{\partial y}\\ =\left(1-2X\right)\left[Y\left(B_{1}-D_{1}+N-\alpha_{1}N\right)+S_{1}-C_{1}\right]+\left(1-2Y\right)\left[X\left(L_{2}-D_{2}-\alpha_{2}N\right)+F_{2}-C_{2}\right]. \end{array}$$

The article "Research on the Behavior Evolution of Interest Groups in Book Reverse Logistics" was published in 2022. Journal: Comput Intell Neurosci.

## 3. Analysis on the Stability of Interest Groups Based on Evolutionary Game

This paper analyzes the evolution process of the strategic system of book publishers and book retailers and combines the replication dynamic equation (4) to obtain five evolutionary equilibrium points of system evolution (0, 0)，(1, 0)，(0, 1)，(1, 1)，(*X*_0_, *Y*_0_), where *X*_0_ = (*C*_2_ − *F*_2_)/(*L*_2_ − *D*_2_ − *α*_2_*N*), *Y*_0_ = (*C*_1_ − *S*_1_)/(*B*_1_ − *D*_1_ + *N* − *α*_1_*N*). If and only if 0 < (*C*_2_ − *F*_2_)/(*L*_2_ − *D*_2_ − *α*_2_*N*) < 1, 0 < (*C*_1_ − *S*_1_)/(*B*_1_ − *D*_1_ + *N* − *α*_1_*N*) < 1, (*X*_0_, *Y*_0_) may be the stable equilibrium point of the system. Since the parameter value range will affect the evolutionary stability strategy of the system, this paper will discuss the stability strategy of the evolutionary system in four cases.

1. Case 1: *β*_1_ >0 , *β*_2_ > 0. Substitute *β*_1_ > 0 and *β*_2_ > 0 into formulas (6) and (7) to obtain the expression of the determinant and trace of the system equilibrium point, as shown in Table 2.
2. To accurately analyze the relationship between book publishers and book retailers participating in the optimization, the parameters are assigned, as shown in Table 3. This paper can get the dynamic evolution path and trend of replication of book publishers and book retailers in Case 1, as shown in Figure 1.
3. It can be seen from Case 1 that when *β*_1_ > 0, *β*_2_ > 0, that is, *B*_1_ − *C*_1_ + *N* − *α*_1_*N* > *D*_1_ − *S*_1_, *L*_2_ − *C*_2_ − *α*_2_*N* > *D*_2_ − *F*_2_, the net revenue of book publishers and book retailers participating in the optimization is greater than the net revenue of not participating in optimization. The two stability policies that exist in the system are related to the initial states of *X* and *Y*. When both parties participate in a low proportion, the system tends to approach the (0, 0) strategy, that is, both parties choose not to participate in optimization. When both parties participate in a high proportion of optimization, the system tends to approach the strategy (1, 1), that is, both parties choose to participate in optimization.
4. Case 2: *β*_1_ < 0, *β*_2_ > 0. In the same way, this paper obtains the expression of the determinant and trace of the equilibrium point of the system, as shown in Table 4.
5. Similarly, the parameters are assigned, as shown in Table 5. This paper can get the dynamic evolution path and trend of replication of book publishers and book retailers in Case 2, as shown in Figure 2.
6. Case 3: *β*_1_ > 0, *β*_2_ < 0. In the same way, this paper obtains the expression of the determinant and trace of the equilibrium point of the system, as shown in Table 6.
7. Similarly, the parameters are assigned, as shown in Table 7. This paper can get the dynamic evolution path and trend of replication of book publishers and book retailers in Case 3, as shown in Figure 3.
8. It can be seen from Case 2 and Case 3 that when *β*_1_ < 0, *β*_2_ > 0 or *β*_1_ > 0, *β*_2_ < 0, that is, *B*_1_ − *C*_1_ + *N* − *α*_1_*N* < *D*_1_ − *S*_1_, *L*_2_ − *C*_2_ − *α*_2_*N* > *D*_2_ − *F*_2_ or *B*_1_ − *C*_1_ + *N* − *α*_1_*N* > *D*_1_ − *S*_1_, *L*_2_ − *C*_2_ − *α*_2_*N* < *D*_2_ − *F*_2_, the net revenue of either book publishers or book retailers participating in optimization is less than the net revenue of not participating in the optimization, both parties will not participate in the optimization, so (0,0) is an evolutionary stability strategy.
9. Case 4: *β*_1_ < 0, *β*_2_ < 0. In the same way, this paper obtains the expression of the determinant and trace of the equilibrium point of the system, as shown in Table 8.

The article "Research on the Behavior Evolution of Interest Groups in Book Reverse Logistics" was published in 2022. Journal: Comput Intell Neurosci.

Similarly, the parameters are assigned, as shown in Table 9. This paper can get the dynamic evolution path and trend of replication of book publishers and book retailers in Case 4, as shown in Figure 4.

It can be seen from Case 4 that when *β*_1_ < 0, *β*_2_ < 0, that is, *B*_1_ − *C*_1_+*N* − *α*_1_*N* < *D*_1_ − *S*_1_, *L*_2_ − *C*_2_ − *α*_2_*N* < *D*_2_ − *F*_2_, the net revenue of book publishers and book retailers participating in the optimization is less than the net revenue of not participating in optimization. Thus, both parties chose not to participate in the optimization strategy.

## 4. Sensitivity Analysis of Group Behavior Evolution System

### 4.1. The Influence of the Initial State on the Evolution Path of the System

By changing the initial state of the proportion of book publishers participating in optimization *X* and the proportion of book retailers participating in optimization *Y*, this paper further analyzed the influence of different proportions of initial states on the evolution path and stability strategy of the system under the condition of Case 1 and obtained the simulation results by using MATLAB software.

#### 4.1.1. The Evolution Path of Book Publishers

1. Discuss the evolution path of book publishers under different proportions of book retailers' selection strategies. It is assumed that when the proportion of book retailers participating in the optimization is selected with a probability of 0.5, the book publishers participate with the probability of 0.1, 0.3, 0.5, 0.7, and 0.9, respectively. The simulation results are shown in Figure 5.
2. Discuss the evolution path of book publishers under different proportions of book publishers' selection strategies. It is assumed that when the proportion of book retailers participating in the optimization is selected with a probability of 0.5, the book publishers participate with the probability of 0.1, 0.3, 0.5, 0.7, and 0.9, respectively. The simulation results are shown in Figure 6.

#### 4.1.2. The Evolutionary Path of Book Retailers

1. Discuss the evolution path of book retailers under different proportions of book publishers' selection strategies. It is assumed that when the proportion of book retailers participating in the optimization is selected with a probability of 0.5, the book publishers participate with the probability of 0.1, 0.3, 0.5, 0.7, and 0.9, respectively. The simulation results are shown in Figure 7.
2. Discuss the evolution path of book retailers under different proportions of book retailers' selection strategies. It is assumed that when the proportion of book publishers participating in the optimization is selected with a probability of 0.5, the book retailers participate with the probability of 0.1, 0.3, 0.5, 0.7, and 0.9, respectively. The simulation results are shown in Figure 8.

As can be seen from Figures 5–8, when the initial proportion of book publishers or book retailers choosing to participate in the optimization is relatively low, for example, when the value is 0.1, 0.3, or 0.5, its evolutionary path tends to the unsatisfactory state of not participating in the optimization. When the initial proportion of book publishers or book retailers choosing to participate in the optimization is relatively high, such as 0.7 or 0.9, its evolutionary path tends to the ideal state of participating in the optimization.

The article "Research on the Behavior Evolution of Interest Groups in Book Reverse Logistics" was published in 2022. Journal: Comput Intell Neurosci.

### 4.2. The Influence of Parameter Value Changes on the Evolutionary Game System

#### 4.2.1. Theoretical Analysis

When the net revenue of book publishers and book retailers participating in the optimization is greater than the net revenue of not participating in the optimization, that is, *β*_1_ > 0, *β*_2_ > 0, the evolutionary system will eventually tend to the (0, 0) strategy that neither side will choose to participate in the optimization or both sides tend to choose (1, 1) strategy that participates in the optimization. Therefore, (0, 0) and (1, 1) are evolutionary stable strategies of the system, and the point *D* (*X*_0_, *Y*_0_) is the saddle point. The specific evolution process is shown in Figure 9.

The regional area of quadrilateral AOCD represents the probability that neither book publishers nor book retailers will participate in the optimization, while the regional area of quadrilateral ABCD represents the probability that both book publishers and book retailers will participate in the optimization. Therefore, the area size of the quadrilateral can represent the possibility that the two sides of the game choose different corresponding strategies, and its size is related to the position of the saddle point (*X*_0_, *Y*_0_). The probability of system stability strategy can be changed by changing the numerical size of the saddle point parameter to guide the evolutionary game system to evolve towards the ideal state, where *X*_0_=(*C*_2_ − *F*_2_)/(*L*_2_ − *D*_2_ − *α*_2_*N*), *Y*_0_=(*C*_1_ − *S*_1_)/(*B*_1_ − *D*_1_+*N* − *α*_1_*N*).

Let *S*_*ABCD*_ represent the area of quadrilateral *ABCD* and *S*_*AOCD*_ represent the area of quadrilateral *AOCD*.

(8) $$\begin{array}{c} S_{ABCD}=1-\frac{1}{2}\left(\frac{C_{2}-F_{2}}{L_{2}-D_{2}-\alpha_{2}N}+\frac{C_{1}-S_{1}}{B_{1}-D_{1}+N-\alpha_{1}N}\right), \end{array}$$

(9) $$\begin{array}{c} S_{AOCD}=\frac{1}{2}\left(\frac{C_{2}-F_{2}}{L_{2}-D_{2}-\alpha_{2}N}+\frac{C_{1}-S_{1}}{B_{1}-D_{1}+N-\alpha_{1}N}\right). \end{array}$$

According to formulas (8) and (9), the parameters in the game model of book publishers-book retailers are analyzed, and Table 10 is obtained.

From Table 10, it can be seen that when the production and sales risk ratio of book publishers decreases and the cost of reverse logistics decreases, the cost of book publishers and book retailers participating in optimization reduces and the revenue increases, and the cost of not participating in optimization reduces and the revenue decreases, and the system will reach the (1, 1) state more quickly. When N reaches condition *X* = 1, the probability of both companies participating in the optimization of book reverse logistics is the greatest.

The article "Research on the Behavior Evolution of Interest Groups in Book Reverse Logistics" was published in 2022. Journal: Comput Intell Neurosci.

#### 4.2.2. Numerical Simulation

To study the influence of parameter values on the evolution path and trend of the system, this paper selects an appropriate initial state, *X* = 0.8, *Y* = 0.8, and changes the values of *α*_1_, *α*_2_, *N*, *B*_1_, *L*_2_, *C*_1_, *C*_2_, *S*_1_, *F*_2_, *D*_1_, and *D*_2_ at the same time. The specific values are shown in Table 11. Group A is the control group, and the other groups are the experimental groups.

1. The influence of *N* changes on the evolution path. Keep other parameters unchanged and change the value of *N* (as shown in *E* in Table 11) to obtain a simulation diagram of the evolution trend of book publishers and book retailers, as shown in Figure 10.
2. It can be seen from Figure 10 that when *N* increases, the proportion of book retailers participating in the optimization greatly decreases, which means that the willingness of book retailers to participate in the optimization decreases, and the convergence speed of the system slows down; the proportion of book publishers participating in the optimization has a small increase, but its impact on the evolution path is too small, so the system will more slowly reach the ideal state where both parties participate in the optimization.
3. The influence of *α*_1_ and *α*_2_ changes on the evolution path. Change the size of *α*_1_ and *α*_2_, keep *α*_1_ + *α*_2_ = 1 and other parameters unchanged, study their influence on the evolutionary system (as shown in *G*_1_ and *G*_2_ in Table 11), and obtain the evolutionary trend simulation diagram of book publishers and book retailers, as shown in Figure 11.
4. It can be seen from Figure 11 that when the production and sales risk ratio of book publishers decreases and the production and sales risk ratio of book retailers increases, it will speed up book publishers to reach the ideal state of participating in the optimization and slow down book retailers that have reached the ideal state of participating in the optimization. Under the condition of the same production and sales risk ratio, the proportion of book publishers participating in the optimization is greater than that of book retailers, indicating that the possibility of book publishers participating in the optimization is greater than the possibility of book retailers participating in the optimization when the production and sales risks are relatively high.
5. The influence of *C*_1_ and *C*_2_ changes on the evolution path. Keep other parameters unchanged and change the values of *C*_1_ and *C*_2_, respectively (as shown in *H*_1_ and *H*_2_ in Table 11), to obtain a simulation diagram of the evolution trend of book publishers and book retailers, as shown in Figure 12.
6. It can be seen from Figure 12 that when the cost of book publishers and book retailers participating in the optimization increases, the revenue of participating in the optimization will decrease, and the willingness to participate in the optimization will decrease, slowing down the speed at which the system converges to the ideal state participating in the optimization. On the contrary, it will increase the revenue of book publishers and book retailers participating in the optimization, increase the willingness to participate in the optimization, and accelerate the speed of convergence.
7. The influence of *S*_1_ and *F*_2_ changes on the evolution path. Keep other parameters unchanged and change the values of *S*_1_ and *F*_2,_ respectively (as shown in *J*_1_ and *J*_2_ in Table 11), to obtain a simulation diagram of the evolution trend of book publishers and book retailers, as shown in Figure 13.
8. As can be seen from Figure 13, when *S*_1_ and *F*_2_ increase, the revenue of book publishers and book retailers not participating in the optimization will decrease, and both sides' willingness to participate in the optimization will be stronger, accelerating the convergence speed of the system and reaching the ideal state of participating in optimization more quickly. On the contrary, the result is the opposite.
9. The influence of *B*_1_ and *L*_2_ changes on the evolutionary path. Keep other parameters unchanged and change the values of *B*_1_ and *L*_2_ respectively (as shown in *K*_1_ and *K*_2_ in Table 11), to obtain a simulation diagram of the evolution trend of book publishers and book retailers, as shown in Figure 14.
10. It can be seen from Figure 14 that when the revenue of book publishers and book retailers participating in the optimization increases, the willingness to participate in the optimization will increase, speeding up the convergence of the system. Conversely, the willingness of book publishers and book retailers to participate in the optimization will decrease, which will slow down the system's convergence speed.
11. The influence of *D*_1_ and *D*_2_ changes on the evolutionary path. Keep other parameters unchanged and change the values of *D*_1_ and *D*_2_, respectively (as shown in *P*_1_ and *P*_2_ in Table 11), to obtain a simulation diagram of the evolution trend of book publishers and book retailers, as shown in Figure 15.

The article "Research on the Behavior Evolution of Interest Groups in Book Reverse Logistics" was published in 2022. Journal: Comput Intell Neurosci.

It can be seen from Figure 15 that when book publishers and book retailers do not participate in the optimization, revenue increases, and book publishers and book retailers will reduce their willingness to participate in the optimization, slowing down system convergence speed. Conversely, the willingness of book publishers and book retailers to participate in the optimization will increase, speeding up system convergence.

## 5. Conclusion

Based on the research of reverse logistics and evolutionary game theory by domestic and foreign scholars, this paper constructs an evolutionary game model between book publishers and book retailers, obtains two evolutionary stable strategies (participation, participation) and (non-participation, non-participation), and uses MATLAB to carry out numerical simulation to analyze the evolution path of the two companies under different evolutionary and stable strategies. The main conclusions are as follows. (1) Through exploring the stability of the interest groups of the evolutionary game in different situations and the influence of the initial state on the evolution path of the system, this paper finds that only when the net revenue of both parties participating in optimization is greater than the net revenue of not participating in optimization, the evolution game system can reach the ideal state where both parties participate in the optimization. When the initial ratio of book publishers and book retailers participating in the optimization is greater than or equal to 0.7, the system will eventually evolve into the ideal state of participating in optimization. (2) Through analyzing the influence of parameter value changes on the evolutionary game system, this paper found that when the cost of participating in the book reverse logistics reaches the condition of (*C*_2_ − *F*_2_)/(*L*_2_ − *D*_2_ − *α*_2_*N*)^2^=(*C*_1_ − *S*_1_)/(*B*_1_ − *D*_1_+*N* − *α*_1_*N*)^2^, the probability of both parties participating in the optimization is the greatest. Under the condition of the same production and sales risk ratio, the proportion of book publishers participating in the optimization is greater than the proportion of book retailers participating in the optimization, indicating that when the production and sales risk ratio is relatively high, the possibility of book publishers participating in the optimization is greater than the possibility of book retailers participating in optimization. When the production and sales risk ratio of book publishers decreases and the cost of reverse logistics decreases, the cost of book publishers and book retailers participating in optimization reduces and the revenue increases, and the cost of not participating in optimization reduces and the revenue decreases, and the system will more quickly reach the ideal state where both parties participate in the optimization.

The article "Research on the Behavior Evolution of Interest Groups in Book Reverse Logistics" was published in 2022. Journal: Comput Intell Neurosci.

## Figures and Tables

**Figure 1:** Evolution path diagram in Case 1. (a) Evolution path of system. (b) Evolution path of book publishers. (c) Evolution path of book retailers.

**Figure 2:** Evolution path diagram in Case 2. (a) Evolution path of system. (b) Evolution path of book publishers. (c) Evolution path of book retailers.

**Figure 3:** Evolution path diagram in Case 3. (a) Evolution path of system. (b) Evolution path of book publishers. (c) Evolution path of book retailers.

**Figure 4:** Evolution path diagram in Case 4. (a) Evolution path of system. (b) Evolution path of book publishers. (c) Evolution path of book retailers.

**Figure 5:** Evolution path when the initial state of *X* is the same.

**Figure 6:** Evolution path when the initial state of *Y* is the same.

**Figure 7:** Evolution path when the initial state of *X* is the same.

**Figure 8:** Evolution path when the initial state of *Y* is the same.

**Figure 9:** Phase diagram of system evolution in Case 1.

**Figure 10:** The simulation diagram of the influence of *N* on the evolution path.

**Figure 11:** The simulation diagram of the influence of *α*_1_ and *α*_2_ on the evolution path.

**Figure 12:** The simulation diagram of the influence of *C*_1_ and *C*_2_ on the evolution path.

**Figure 13:** The simulation diagram of the influence of *S*_1_ and *F*_2_ on the evolution path.

**Figure 14:** The simulation diagram of the influence of *B*_1_ and *L*_2_ on the evolution path.

**Figure 15:** The simulation diagram of the influence of *D*_1_ and *D*_2_ on the evolution path.

**Table 1:** Matrix of payment.

Game subject		Book retailers	
		Participation (*Y*)	Non-participation (1 − *Y*)
Book publishers	Participation (*X*)	*B *_1_–*C*_1_–*α*_1_*N*, *L*_2_–*C*_2_–*α*_2_*N*	*D *_1_–*C*_1_–*N*, *D*_2_–*F*_2_
	Non-participation (1 − *X*)	*D *_1_–*S*_1_–*N*, *D*_2_–*C*_2_	*D *_1_–*S*_1_–*N*, *D*_2_–*F*_2_

**Table 2:** The local stability of the equilibrium point in Case 1.

Equilibrium point	det (*J*)	tr (*J*)	Local stability	Strategy profile
(0, 0)	+	−	ESS	(Non-participation, non-participation)
(1, 0)	+	Uncertain	Unstable point	(Participation, non-participation)
(0, 1)	+	Uncertain	Unstable point	(Non-participation, participation)
(1, 1)	+	−	ESS	(Participation, participation)
(*X*_0_, *Y*_0_)	−	0	Saddle point	

The article "Research on the Behavior Evolution of Interest Groups in Book Reverse Logistics" was published in 2022. Journal: Comput Intell Neurosci.

**Table 3:** Assignment of each parameter in Case 1.

Parameter	*α*_1_	*α*_2_	*N*	*C*_1_	*C*_2_	*S*_1_	*F*_2_	*B*_1_	*L*_2_	*D*_1_	*D*_2_
Assignment	0.5	0.5	20	17	24	10	11	15	50	10	20

**Table 4:** The local stability of the equilibrium point in Case 2.

Equilibrium point	det (*J*)	tr (*J*)	Local stability	Strategy profile
(0, 0)	+	−	ESS	(Non-participation, non-participation)
(0, 1)	−	Uncertain	Saddle point	(Participation, non-participation)
(1, 0)	+	+	Unstable point	(Non-participation, participation)
(1, 1)	−	Uncertain	Saddle point	(Participation, participation)
(*X*_0_, *Y*_0_)	+	0	Unstable point	

**Table 5:** Assignment of each parameter in Case 2.

Parameter	*α*_1_	*α*_2_	*N*	*C*_1_	*C*_2_	*S*_1_	*F*_2_	*B*_1_	*L*_2_	*D*_1_	*D*_2_
Assignment	0.5	0.5	20	22	24	4	11	15	45	10	20

**Table 6:** The local stability of the equilibrium point in Case 3.

Equilibrium point	det (*J*)	tr (*J*)	Local stability	Strategy profile
(0, 0)	+	−	ESS	(Non-participation, non-participation)
(0, 1)	+	+	Unstable point	(Participation, non-participation)
(1, 0)	−	Uncertain	Saddle point	(Non-participation, participation)
(1, 1)	−	Uncertain	Saddle point	(Participation, participation)
(*X*_0_, *Y*_0_)	+	0	Unstable point	

**Table 7:** Assignment of each parameter in Case 3.

Parameter	*α*_1_	*α*_2_	*N*	*C*_1_	*C*_2_	*S*_1_	*F*_2_	*B*_1_	*L*_2_	*D*_1_	*D*_2_
Assignment	0.5	0.5	20	22	24	10	11	15	32	10	20

**Table 8:** The local stability of the equilibrium point in Case 4.

Equilibrium point	det (*J*)	tr (*J*)	Local stability	Strategy profile
(0, 0)	+	−	ESS	(Non-participation, non-participation)
(0, 1)	−	Uncertain	Saddle point	(Participation, non-participation)
(1, 0)	−	Uncertain	Saddle point	(Non-participation, participation)
(1, 1)	+	+	Unstable point	(Participation, participation)
(*X*_0_, *Y*_0_)	−	0	Saddle point	

**Table 9:** Assignment of each parameter in Case 4.

Parameter	*α*_1_	*α*_2_	*N*	*C*_1_	*C*_2_	*S*_1_	*F*_2_	*B*_1_	*L*_2_	*D*_1_	*D*_2_
Assignment	0.5	0.5	20	22	24	4	11	15	32	10	20

**Table 10:** Influence of parameter changes on evolution stability results.

Variation of parameters	Basis of judgment	Result
*α*_1_↑	∂*S*_*ABCD*_/∂*α*_1_=−(*N*(*C*_1_ − *S*_1_))/(2(*B*_1_ − *D*_1_+*N* − *α*_1_*N*)^2^) < 0, ∂*S*_*ABCD*_/∂*α*_1_=(*N*(*C*_1_ − *S*_1_))/(2(*B*_1_ − *D*_1_+*N* − *α*_1_*N*)^2^) > 0	Both parties prefer not to participate in the optimization, and the evolutionary game system converges to the point (0, 0).
*α*_2_↑	∂*S*_*ABCD*_/∂*α*_2_=−(*N*(*C*_2_ − *F*_2_))/(2(*L*_2_ − *D*_2_ − *α*_2_*N*)^2^) < 0, ∂*S*_*ABCD*_/∂*α*_2_=(*N*(*C*_2_ − *F*_2_))/(2(*L*_2_ − *D*_2_ − *α*_2_*N*)^2^) > 0	
*D*_1_↑	∂*S*_*ABCD*_/∂*D*_1_=−(*C*_1_ − *S*_1_)/(2(*B*_1_ − *D*_1_+*N* − *α*_1_*N*)^2^) < 0, ∂*S*_*AOCD*_/∂*D*_1_=(*C*_1_ − *S*_1_)/(2(*B*_1_ − *D*_1_+*N* − *α*_1_*N*)^2^) > 0	
*D*_2_↑	∂*S*_*ABCD*_/∂*D*_2_=−(*C*_2_ − *F*_2_)/(2(*L*_2_ − *D*_2_ − *α*_2_*N*)^2^) < 0, ∂*S*_*AOCD*_/∂*D*_2_=(*C*_2_ − *F*_2_)/(2(*L*_2_ − *D*_2_ − *α*_2_*N*)^2^) > 0	
*C*_1_↑	∂*S*_*ABCD*_/∂*C*_1_=−*C*_1_/(2(*B*_1_ − *D*_1_+*N* − *α*_1_*N*)) < 0, ∂*S*_*AOCD*_/∂*C*_1_=*C*_1_/(2(*B*_1_ − *D*_1_+*N* − *α*_1_*N*)) > 0	
*C*_2_↑	∂*S*_*ABCD*_/∂*C*_2_=−*C*_2_/(2(*L*_2_ − *D*_2_ − *α*_2_*N*)) < 0, ∂*S*_*AOCD*_/∂*C*_2_=*C*_2_/2(*L*_2_ − *D*_2_ − *α*_2_*N*) > 0	
*S*_1_↑	∂*S*_*ABCD*_/∂*S*_1_=*S*_1_/2(*B*_1_ − *D*_1_+*N* − *α*_1_*N*) > 0, ∂*S*_*AOCD*_/∂*S*_1_=−*S*_1_/(2(*B*_1_ − *D*_1_+*N* − *α*_1_*N*)) < 0	Both parties are more inclined to participate in the optimization, and the evolutionary game system converges to the point (1, 1).
*F*_2_↑	∂*S*_*ABCD*_/∂*F*_2_=*F*_2_/(2(*L*_2_ − *D*_2_ − *α*_2_*N*)) > 0, ∂*S*_*AOCD*_/∂*F*_2_=−*F*_2_/(2(*L*_2_ − *D*_2_ − *α*_2_*N*)) < 0	
*B*_1_↑	∂*S*_*ABCD*_/∂*B*_1_=*C*_1_ − *S*_1_/(2(*B*_1_ − *D*_1_+*N* − *α*_1_*N*)^2^) > 0, ∂*S*_*AOCD*_/∂*B*_1_=−*C*_1_ − *S*_1_/(2(*B*_1_ − *D*_1_+*N* − *α*_1_*N*)^2^) < 0	
*L*_2_↑	∂*S*_*ABCD*_/∂*L*_2_=(*C*_2_ − *F*_2_)/(2(*L*_2_ − *D*_2_ − *α*_2_*N*)^2^) > 0, ∂*S*_*AOCD*_/∂*L*_2_=−(*C*_2_ − *F*_2_)/(2(*L*_2_ − *D*_2_ − *α*_2_*N*)^2^) < 0	
N	当 *C*_2_ − *F*_2_/(*L*_2_ − *D*_2_ − *α*_2_*N*)^2^=*C*_2_ − *F*_2_/(*B*_1_ − *D*_1_+*N* − *α*_1_*N*)^2^ 时	Both book publishers and book retailers have the greatest probability of participating in the optimization.

The article "Research on the Behavior Evolution of Interest Groups in Book Reverse Logistics" was published in 2022. Journal: Comput Intell Neurosci.

**Table 11:** Parameter values.

Parameter	*α*_1_	*α*_2_	*N*	*C*_1_	*C*_2_	*S*_1_	*F*_2_	*B*_1_	*L*_2_	*D*_1_	*D*_2_
*A*	0.5	0.5	20	17	24	10	11	15	50	10	20
*E*	0.5	0.5	30	17	24	10	11	15	50	10	20
*G*_1_	0.8	0.2	20	17	24	10	11	15	50	10	20
*G*_2_	0.3	0.7	20	17	24	10	11	15	50	10	20
*H*_1_	0.5	0.5	20	22	24	10	11	15	50	10	20
*H*_2_	0.5	0.5	20	17	19	10	11	15	50	10	20
*J*_1_	0.5	0.5	20	17	24	5	11	15	50	10	20
*J*_2_	0.5	0.5	20	17	24	10	16	15	50	10	20
*K*_1_	0.5	0.5	20	17	24	10	11	25	50	10	20
*K*_2_	0.5	0.5	20	17	24	10	11	15	60	10	20
*P*_1_	0.5	0.5	20	17	24	10	11	15	50	5	20
*P*_2_	0.5	0.5	20	17	24	10	11	15	50	10	15

## Data Availability

The data for all Figures used to support the findings of this study are included within the article.
